The article "Prediction of Prognosis and Molecular Mechanism of Ferroptosis in Hepatocellular Carcinoma Based on Bioinformatics Methods" was retracted in 2023. Reasons: signs of a paper mill; suspected computer-generated content; unreliable results or conclusions; concerns about the data.

# Prediction of Prognosis and Molecular Mechanism of Ferroptosis in Hepatocellular Carcinoma Based on Bioinformatics Methods

**DOI:** 10.1155/2022/4558782

**Published:** 2022-06-21

**Authors:** Yuanpeng Xiong, Yonghao Ouyang, Kang Fang, Gen Sun, Shuju Tu, Wanpeng Xin, Yongyang Wei, Weidong Xiao

**Affiliations:** Department of General Surgery, The First Affiliated Hospital of Nanchang University, Nanchang 330006, China

## Abstract

**Background:**

As an iron-dependent type of programmed cell death, ferroptosis plays an important role in the pathogenesis and progression of hepatocellular carcinoma (HCC). Long noncoding RNAs (lncRNAs) have been linked to the prognosis of patients with HCC in a number of studies. Nevertheless, the predictive value of lncRNAs (FRLs) associated with ferroptosis in HCC has not been fully elucidated.

**Methods:**

Download RNA sequencing data and clinical profiles of HCC patients from The Cancer Genome Atlas (TCGA) database. The FRLs associated with prognosis were determined by Pearson's correlation analysis. After that, prognostic signature for FRLs was established using Cox and LASSO regression analyses. Meanwhile, survival analysis, correlation analysis of clinicopathological features, Cox regression, receiver operating characteristic (ROC) curve, and nomogram were used to analyze the FRL signature's predictive capacity. The relationship between signature risk score, immune cell infiltration, and chemotherapy drug sensitivity is further studied.

**Results:**

In total, 93 FRLs were found to be of prognostic value in patients with HCC. A five-FRL signature comprising AC015908.3, LINC01138, AC009283.1, Z83851.1, and LUCAT1 was created in order to enhance the prognosis prediction with HCC patients. The signature demonstrated a good predictive potency, according to the Kaplan-Meier and ROC curves. The five-FRL signature was found to be a risk factor independent of various clinical factors using Cox regression and stratified survival analysis. The high-risk group was shown to be enriched in tumorigenesis and immune-related pathways according to GSEA analysis. Additionally, immune cell infiltration, immune checkpoint molecules, and half-inhibitory concentrations differed considerably between risk groups, implying that this signature could be used to evaluate the clinical efficacy of chemotherapy and immunotherapy.

**Conclusion:**

The five-FRL risk signature is helpful for assessing the prognosis of HCC patients and improving therapy options, so it can be further applied clinically.

## 1. Introduction

Liver cancer is currently the sixth most common malignant tumor known, and its incidence and mortality are annually rising over the worldwide [1]. Hepatocellular carcinoma (HCC) represents the major histologic subtype of liver cancer, accounting for around 75% of all cases. Hepatitis virus infection, aflatoxin exposure, alcoholic cirrhosis, diabetes, and smoking are considered as major risk factors for HCC, and the incidence is higher in men than in women [2]. Hepatectomy, liver transplantation, thermal ablation, transarterial chemoembolization (TACE), hepatic arterial infusion chemotherapy (HAIC), targeted therapy, and immunotherapy are currently the most common treatments for HCC [3, 4]. Despite the continuous improvement of treatment methods, the overall prognosis of HCC remains unsatisfactory. Furthermore, there are no effective prognostic indicators for HCC. Although serum alpha-fetoprotein (AFP) was commonly used to diagnose and predict the prognosis of HCC, its clinical application is greatly compromised by the presence of many AFP-negative patients (AFP < 20 ng/mL) [5]. As a result, the search for up-to-date and reliable biomarkers is crucial to predict HCC prognosis.

The article "Prediction of Prognosis and Molecular Mechanism of Ferroptosis in Hepatocellular Carcinoma Based on Bioinformatics Methods" was retracted in 2023. Reasons: signs of a paper mill; suspected computer-generated content; unreliable results or conclusions; concerns about the data.

Ferroptosis is a newly defined nonapoptotic programmed cell death mechanism that relies on iron and is triggered by fatal lipid peroxidation. It differs from other types of cell death such as apoptosis, autophagy, and pyroptosis [6, 7]. Ferroptosis appears to play a role in the development of a variety of liver diseases, including alcoholic liver disease, nonalcoholic fatty liver disease, viral hepatitis, liver cirrhosis, and HCC [8, 9]. Importantly, ferroptosis has potential functions in inhabiting tumor progression and metastasis and restricting drug resistance in HCC. With the extensive research into the mechanisms of ferroptosis, a number of ferroptosis-related genes (FRGs) involved in this process have been identified in HCC, although there are inconsistencies on their functions [10–12]. Recently, a five-FRG (G6PD, HMOX1, LOX, SLC7A11, and STMN1) signature had been established for prognostic model for HCC patients, and the areas under the ROC curve (AUC) for 5-year overall survival (OS) was 0.756 [12].

Long noncoding RNAs (lncRNAs) are a type of noncoding RNA with a length of more than 200 nucleotides that can affect gene expression via posttranscriptional regulatory mechanisms and play a role in a number of biological processes [13]. The functions of lncRNA can be better evaluated by lncRNA-mRNA coexpression analysis [14]. The onset, progression, and prognosis of HCC are all linked to aberrant lncRNA expression [15, 16]. Moreover, earlier research has shown that lncRNAs can regulate the expression of FRGs in HCC [17]. lncRNA GABPB1-AS1, for example, promotes erastin-induced ferroptosis in HCC by suppressing GABPB1 expression, lowering cellular antioxidant capability and cell viability [18]. Therefore, ferroptosis-related lncRNAs (FRLs) could be valuable in predicting prognosis and serving as targets for treatment of HCC.

The article "Prediction of Prognosis and Molecular Mechanism of Ferroptosis in Hepatocellular Carcinoma Based on Bioinformatics Methods" was retracted in 2023. Reasons: signs of a paper mill; suspected computer-generated content; unreliable results or conclusions; concerns about the data.

FRLs associated with HCC prognosis were screened on RNA sequencing data from The Cancer Genome Atlas (TCGA) database. The study then used multivariate Cox and LASSO regression analyses to create a five-FRL signature for predicting the survival of HCC patients. Its predictive value was further validated by internal verification (TCGA cohorts), external verification (GEO cohorts), and principal component analysis (PCA). Subsequently, the signature's putative biological role was investigated using functional enrichment analysis. In addition, we looked into the relationship between immune cell infiltration, chemotherapeutic drug sensitivity, and the five-FRL signature. These findings might provide new insights into the prognostication and treatment of HCC.

## 2. Materials and Methods

### 2.1. Data Collection

The RNA sequencing (RNA-seq) data and corresponding clinical data of 424 samples (374 samples of HCC tissue and 50 samples of normal hepatic tissues) were downloaded from TCGA database up to February 1, 2022 (https://portal.gdc.cancer.gov/repository). The patients with a survival time of <30 days and missing expression data were excluded, leaving 343 HCC samples in the final cohort. Supplementary Table S1 shows the 259 FRGs that were obtained from the FerrDb database (http://www.zhounan.org/ferrdb). The clinical information and gene expression profile data of 115 HCC patients were obtained from the GEO database (GSE76427, https://www.ncbi.nlm.nih.gov/geo/) as the external verification cohort.

### 2.2. Identification of Differentially Expressed FRGs

FRG expression data were filtered from the TCGA data. The “limma” package of R software (version 4.1.0) was then used to examine differentially expressed genes between tumor and normal tissues. Differentially expressed FRGs (DEFRGs) were identified according to false discovery rate (FDR) < 0.05 and |log2FC| > 1.

### 2.3. Construction and Validation of a FRL Signature

Pearson's correlation analysis was used to look at the coexpression correlations between DEFRGs and lncRNAs in HCC samples, with a coefficient |*R*^2^| > 0.3 and *P* < 0.001 cutoff. To find the prognosis-related lncRNAs, we used univariate Cox (UniCox) regression analysis. The ideal panel of prognostic lncRNAs and an optimal signature were then determined using LASSO and multivariate Cox (multiCox) regression analyses. The standardized expression levels of each risk lncRNA and its matching regression coefficient were then used to calculate each patient's survival risk score. The calculation was as follows: risk score = ∑Coef_lncRNA_ × Exp_lncRNA_), where Coef_lncRNA_ and Exp_lncRNA_ represent the regression coefficient and the expression of lncRNA, respectively. The patients were then separated into high- and low-risk groups according to the median risk score value. The Kaplan-Meier survival curves were created with R software, and the log-rank test was used to examine the survival differences between the two groups. The time-dependent ROC curve was utilized to evaluate survival prediction; the AUC was calculated to determine the predictive accuracy and specificity of the FRL signature. Additionally, “Scatterplot3d” package was used for the principal component analysis (PCA) to test the clustering ability of the signature. On the independent prognostic factor of HCC, UniCox and multiCox proportional hazard regression analyses for OS were conducted. Furthermore, the nomogram was created with the risk score and other clinicopathological features, and its accuracy is verified by the calibration curve. To ensure the signature's stability, we randomly divide the TCGA dataset patients into two cohorts as internal verification and then recruit the GEO dataset as external verification. The FRL signature is calculated using data from the entire TCGA cohort, and survival analysis and COX regression analysis were conducted to see if the signature is substantially correlated with OS in each verification cohort. Meanwhile, the ROC curve was developed to evaluate the accuracy of this new model in predicting patient's survival.

The article "Prediction of Prognosis and Molecular Mechanism of Ferroptosis in Hepatocellular Carcinoma Based on Bioinformatics Methods" was retracted in 2023. Reasons: signs of a paper mill; suspected computer-generated content; unreliable results or conclusions; concerns about the data.

### 2.4. Functional Enrichment Analysis

The Kyoto Encyclopedia of Genes and Genomes (KEGG) and Gene Ontology (GO) analyses were conducted using the gene set enrichment analysis (GSEA) software (version 4.10) to clarify the mainly enriched pathways in the high- and low-risk groups. Nominal *P* < 0.05 and FDR < 0.25 were chosen as statistical significance thresholds.

### 2.5. Immune Infiltration Analysis of the FRL Signature

Single-sample gene set enrichment analysis (ssGSEA) was used to calculate the infiltration scores of 16 immune cells and the activity of 13 immune-related pathways. Meanwhile, there was a link between the risk score and immunological checkpoints.

### 2.6. Chemotherapy Drug Sensitivity Analysis of the FRL Signature

Further assessment of chemotherapeutic drug responsiveness in patients with HCC in risk subgroups, the half-maximal inhibitory concentration (IC_50_) of chemotherapy drugs commonly used in clinical treatment of HCC was calculated using the “pRRophetic” package (contains 138 chemotherapy drugs), and differences in IC_50_ values between risk subgroups were analyzed using the Wilcoxon signed-rank test. Statistical significance was defined as *P* value < 0.05.

The article "Prediction of Prognosis and Molecular Mechanism of Ferroptosis in Hepatocellular Carcinoma Based on Bioinformatics Methods" was retracted in 2023. Reasons: signs of a paper mill; suspected computer-generated content; unreliable results or conclusions; concerns about the data.

## 3. Results

### 3.1. Identification of DEFRGs

Figure 1 shows the flowchart for this research. A total of 84 DEFRGs were identified through differential analysis of the RNA-seq data from TCGA. Compared with the normal liver tissues, the expression of 13 DEFRGs (HAMP, MT1G, NNMT, PTGS2, ZFP36, IL6, GLS2, ALB, TUBE1, ATF3, STEAP3, DUSP1, and PLIN2) was downregulated, and 71 DEFRGs (FTL, SLC7A5, FTH1, NRAS, CAV1, NCF2, FADS2, BAP1, PML, HSPA5, DDIT4, ENPP2, DNAJB6, ZNF419, EMC2, AKR1C1, YY1AP1, EGLN2, GPX2, ALOX12, NF2, CS, MAPK3, SLC1A4, AIFM2, HSF1, NOX1, DDIT3, MYB, TFRC, HRAS, ZFP69B, AKR1C2, TAZ, SLC1A5, RPL8, SQSTM1, ABCC1, SLC2A6, SLC38A1, SRC, SLC2A1, TP63, CAPG, SLC2A14, MAFG, SRXN1, NOS2, TXNRD1, NOX5, ALOX15, AKR1C3, HSPB1, ASNS, PRKAA2, ACSL4, DRD4, STMN1, FANCD2, DUOX1, HELLS, G6PD, AURKA, NOX4, ALOX15B, RRM2, CDKN2A, MIOX, MT3, SLC7A11, and NQO1) were upregulated in HCC tissues. The expression of these DEFRGs in tumor and normal tissues using volcano plots, boxplots, and heatmaps were shown in Figures 2(a)–2(c). To further explore the potential biological functions and pathways related to DEFRGs, we carried out further KEGG and GO analyses of the 84 DEFRGs. As we expected, these DEFRGs were mainly enriched in ferroptosis-associated pathways and other cancer-associated pathways (Supplementary Figure 1).

### 3.2. Construction of the FRL Prognostic Signature

There were 764 lncRNAs identified to have a correlation with these 84 DEFRGs in total, considered as FRLs (Supplementary Table S2). UniCox analysis demonstrated that 93 FRLs were associated with the prognosis of HCC (Supplementary Table S3). LASSO regression and multiCox analysis kept five candidate prognostic FRLs (AC015908.3, LINC01138, AC009283.1, Z83851.1, and LUCAT1) after filtration. The expression of these five FRLs in HCC patients was shown in Figure 3(a). To better visualize the five FRLs, we employ Cytoscape and R software. A total of 34 pairings of lncRNA-mRNA in the coexpression network (Figure 3(b); ∣*R*^2^ | >0.3 and *P* < 0.001). In detail, eight FRGs (CS, SLC38A1, MAPK3, ASNS, MAFG, STMN1, RRM2, and FANCD2) had coexpressive connection with AC015908.3; nine FRGs (G6PD, HRAS, MAPK3, CDKN2A, YY1AP1, SLC2A6, STMN1, FANCD2, and HELLS) had coexpressive connection with LINC01138; AC034236.2 was coexpressed with ZNF419; three FRGs (RPL8, GPX2, and HSF1) had coexpressive connection with Z83851.1; thirteen FRGs (G6PD, TXNRD1, SRXN1, GPX2, SLC7A11, FTL, MAFG, FT AC009283H1, AKR1C1, AKR1C2, AKR1C3, SQSTM1, and NQO1) had coexpressive connection with LUCAT1. AC009283.1 and AC015908.3 were protective factors, while Z83851.1, LINC01138, and LUCAT1 were risk factors for prognosis (Figure 3(c)). The expression levels of these five FRLs and their weighting coefficients were used to calculate the risk score of HCC patients. The formula was as follows: risk score = (−0.463 × AC015908.3 expression) + (0.745 × LINC01138 expression) + (−0.916 × AC009283.1 expression) + (0.576 × Z83851.1 expression) + (0.845 × LUCAT expression). The median risk score value (0.898) was used to separate 343 patients with HCC from the TCGA into high-risk (*n* = 170) and low-risk (*n* = 173) groups. The expression outlines of these five FRLs in different risk subgroups were depicted using heatmaps. Two protective lncRNAs were downregulated in the high-risk groups, while 3 risk lncRNAs were upregulated (Figure 3(d)). The Kaplan-Meier curves demonstrated significantly lower OS in the high-risk group (Figures 3(e)–3(g)). The AUC for 1-, 3-, and 5-year OS was 0.768, 0.714, and 0.738, respectively (Figure 3(h)).

The article "Prediction of Prognosis and Molecular Mechanism of Ferroptosis in Hepatocellular Carcinoma Based on Bioinformatics Methods" was retracted in 2023. Reasons: signs of a paper mill; suspected computer-generated content; unreliable results or conclusions; concerns about the data.

### 3.3. Independent Prognostic Analysis and Nomogram Construction

The relationship between risk score, risk lncRNAs, and clinicopathological variables was investigated to determine the five-FRL signature's independent prognostic value, as shown in Table 1 and Figure 4. For the risk score, it was significantly correlated with survival outcome (*P* = 0.002) and tumor N stage (*P* = 0.017) (Figures 4(a) and 4(b)). For FRLs, AC015908.3 was significantly correlated with survival outcome (*P* = 1.133e − 06), gender (*P* = 0.019), tumor stage (*P* = 1.222e − 04), and tumor T stage (*P* = 4.68e − 04) (Figures 4(c)–4(f)); LINC01138 was significantly correlated with survival outcome (*P* = 0.002) and grade (*P* = 0.002) (Figures 4(g) and 4(h)); LUCAT1 was significantly correlated with survival outcome (*P* = 0.034), gender (*P* = 0.010), tumor M stage (*P* = 0.001), and tumor N stage (*P* = 5.975e − 04) (Figures 4(i)–4(l)). According to UniCox analysis, tumor stage, tumor T stage, tumor M stage, and risk score were considered to be significantly prognostic factors (Figure 4(m)). Furthermore, in multiCox analysis, the risk score was considered the only independent prognostic factor (Figure 4(n)). The AUC value of risk score was 0.778, which was markedly higher than that of age, gender, grade, tumor stage, tumor T stage, tumor N stage, and tumor M stage (Figure 4(o)). The five-FRL signature was found to be superior to clinicopathological parameters in predicting HCC patient survival.

To assess the clinical utility of the signature, we created a nomogram involving clinicopathological factors and risk scores. Thus, we assessed and quantified the probability of survival of HCC patients after 1, 3, and 5 years (Figure 5(a)). Meanwhile, the calibration curves revealed an excellent match between the actual OS and the expected OS of 1, 3, and 5 years (Figures 5(b)–5(d)). These results suggested that the five-FRL signature-based nomogram had great clinical utility in predicting the prognosis of HCC patients.

The article "Prediction of Prognosis and Molecular Mechanism of Ferroptosis in Hepatocellular Carcinoma Based on Bioinformatics Methods" was retracted in 2023. Reasons: signs of a paper mill; suspected computer-generated content; unreliable results or conclusions; concerns about the data.

### 3.4. Internal and External Validation of the Five-FRL Prognostic Signature

In order to confirm the five-FRL signature's stability. 343 HCC patients were randomly divided into two cohorts (*n*1 = 171 and *n*2 = 172). The patients' characteristics in the two cohorts were shown in Table 2. According to the findings, patients in the high-risk group had considerably lower OS in both cohorts (Figures 6(a) and 6(b)), which was consistent with the whole dataset's findings. The 1-, 3-, and 5-year survival rates of the two cohorts were 0.818, 0.738, and 0.790 and 0.748, 0.680, and 0.715, respectively (Figures 6(c) and 6(d)). Furthermore, it is impossible to retrieve the other datasets that simultaneously report the five-FRL expression levels, clinical features, and survival status of HCC patients. As a result, the external verification cohort was selected from the GEO dataset (GSE7642), and it contains the expression levels of mRNAs coexpressed with the five FRLs and the survival data of 115 HCC patients. The Kaplan-Meier analysis revealed that the OS of high-risk patients was significantly shorter (*P* = 0.004) (Figure 7(a)). The AUC for 1-, 3-, and 5-year survival rates was 0.798, 0.734, and 0.839, respectively (Figure 7(b)). According to all of the findings, the five-FRL signature had good prognostic power in HCC patients.

### 3.5. Principal Components Analysis (PCA)

The ability of the developed model to cluster the distribution of patients in the risk subgroup population was further evaluated. PCA was used to depict the patient distribution based on the whole genome, FRG sets, FRLs, and predictive signature. The signature was the best for patients, as demonstrated in Figures 8(a)–8(d). Signatures could assign patients with high- and low-risk scores in different quadrants.

### 3.6. Functional Enrichment Analysis

To investigate the five FRLs' potential biological function, GSEA analysis was performed to identify differential enrichment pathways between different risk subgroups. As shown in Figure 9, the high-risk group was primarily enriched in the metabolic pathways associated with ferroptosis: glutathione metabolism; tumor forming pathway: pathways in cancer; and other immune-related pathways: Vibrio cholerae infection, pathogenic Escherichia Coli infection, mTOR signaling pathway, and Leishmania infection. According to the findings, tumor-related and immune-related pathways were overrepresented in high-risk patients.

The article "Prediction of Prognosis and Molecular Mechanism of Ferroptosis in Hepatocellular Carcinoma Based on Bioinformatics Methods" was retracted in 2023. Reasons: signs of a paper mill; suspected computer-generated content; unreliable results or conclusions; concerns about the data.

### 3.7. The Importance of the Five-FRL Signature in Tumor Immune Microenvironment (TIM)

Because of the importance of immune infiltrating cells in TIM, we conducted ssGSEA enrichment scores on several immune cell subsets and associated functions to analyze the relationship between risk scores and immune infiltrating cells and their functions. For immune cells, the findings revealed that activated dendritic cells (aDCs), macrophages, and regulatory T cells (Tregs) were more abundant in the high-risk group, while B cells and mast cells were more abundant in the low-risk group (*P* < 0.05; Figure 10(a)). For the functions of immune cells, the findings revealed that the major histocompatibility complex (MHC) class I score was higher in the high-risk group, while the type II IFN response was lower (*P* < 0.05; Figure 10(b)). These findings suggested that the predictive signature could play a role in TIM by acting on immune infiltrating cells. Since immunological checkpoints play a very important role in immunotherapy, we further analyzed the expression of immune checkpoints in different risk subgroups. The results showed that there were significant differences in 21 immune checkpoints: TNFSF18, TNFRSF18, TNFSF4, TNFSF9, CD86, CD80, TNFRSF8, TNFRSF4, HAVCR2, CD70, VTCN1, TNFRSF9, CD276, LAIR1, HHLA2, TMIGD2, CD44, CD40, TNFRSF14, LGALS9, and CTLA4 (*P* < 0.05; Figure 10(c)). The results suggested that immune checkpoint genes were upregulated in high-risk HCC patients, which facilitated immune evasion and led to poor prognosis.

### 3.8. The Importance of the Five-FRL Signature in Chemotherapy

The significance of the five-FRL signature in predicting chemotherapy drugs' sensitivity to HCC was also assessed. Among these 138 chemotherapeutic drugs, the response to 90 anticancer medicines between two risk subgroups was not statistically significant, and there was a significant difference in the response to 48 anticancer drugs (supplement Table S4). We selected 10 chemotherapy drugs with significant differences and applications in HCC for visualization. The results showed that the IC_50_ of dasatinib, docetaxel, erlotinib, gefitinib, lapatinib, and methotrexate was markedly higher in the high-risk group (Figures 11(a)–11(f)). Cisplatin, gemcitabine, imatinib, and paclitaxel had markedly lower IC_50_ in the high-risk group (Figures 11(g)–11(j)). This indicated that patients in the high-risk group had a better response to the chemotherapeutic drugs cisplatin, gemcitabine, imatinib, and paclitaxel.

## 4. Discussion

As bioinformatics technology has advanced in recent years, a variety of lncRNA-related signatures have been established to predict the outcome of patients with fatal malignancies such as pancreatic cancer, breast cancer, colorectal cancer, and bladder cancer [19–22]. Nevertheless, FRL signatures for forecasting the survival and molecular characteristics of HCC are rarely reported.

The article "Prediction of Prognosis and Molecular Mechanism of Ferroptosis in Hepatocellular Carcinoma Based on Bioinformatics Methods" was retracted in 2023. Reasons: signs of a paper mill; suspected computer-generated content; unreliable results or conclusions; concerns about the data.

Previous research has indicated that various lncRNAs are abnormally expressed and have oncogenic or tumor suppressive roles in HCC [23, 24]. Additionally, lncRNAs play a crucial function in regulating ferroptosis. For example, ZFAS1 facilitates the conversion of lung fibroblasts into myofibroblasts and ferroptosis via acting as a competitive endogenous RNA (ceRNA) through the miR-150-5p/SLC38A1 axis [25]. LINC00336 suppresses ferroptosis in lung cancer by serving as a ceRNA for miR-6852 [26]. lncRNA RP11-89 suppresses ferroptosis through the miR-129-5p/PROM2 axis and contributes to the advancement of bladder cancer [27]. Recently, several FRL signatures with 3-9 lncRNAs have been constructed for the prognosis of HCC, and the AUC for 3-year OS was 0.649-0.812 [17, 28–32] (Table 3). In the present study, we noticed that 84 FRGs were expressed differently in HCC tissues than in normal tissues. Meanwhile, a total of 93 FRLs was identified to be linked to the prognosis of HCC patients. Moreover, five FRLs (AC015908.3, LINC01138, AC009283.1, Z83851.1, and LUCAT1) were identified by UniCox, multiCox, and LASSO regression analysis, based on which a prognostic risk signature was constructed.

This five-FRL signature had a more stable predictive efficiency in both the training cohort and the testing cohort. Among them, LUCAT1 has been shown to directly sponge the onco-miR-181d-5p, and its upregulation is linked to a reduced risk of HCC recurrence [28, 32, 33]. AC015908.3 has been demonstrated to have a certain predictive value in the current model for predicting liver cancer prognosis [31, 34]. Although LINC01138 could boost the invasion and metastasis of HCC cells by activating PRMT5 [35], it was a risk factor in an autophagy-related lncRNA prognosis prediction model of liver cancer [36]. Its role and mechanism of ferroptosis in HCC have not been reported. AC009283.1 was reported as a regulatory of genes involved in proliferation, cell cycle, and apoptosis of breast cancer cells [37] and may be utilized as one of the relevant indicators to forecast the outcome of colon cancer patients [38]. However, the role of AC009283.1 in HCC remains unknown. It is worth noting that there is no related research on Z83851.1. In the current study, Z83851.1 was demonstrated to have a close coexpression relationship with FRGs and have prognostic value for HCC. At the same time, mRNAs with significant coexpression relationship with these five FRLs were found in the current study, including CS, SLC38A1, MAPK3, ASNS, MAFG, STMN1, RRM2, FANCD2, G6PD, HRAS, CDKN2A, YY1AP1, SLC2A6, HELLS, ZNF419, RPL8, GPX2, HSF1, TXNRD1, SRXN1, SL C7A11, FTL, FTH1, AKR1C2, AKR1C3, SQSTM1, and NQO1. These genes have been demonstrated to play key roles in promoting or suppressing ferroptosis. For example, SLC38A1 promotes ferroptosis by regulating glutamine catabolism [39]. YY1AP1 promotes ferroptosis through NF2-YAP signal transduction [40]. NQO1 inhibits ferroptosis in HCC cells by participating in the P62-KEAP1-NRF2 pathway [10].

The article "Prediction of Prognosis and Molecular Mechanism of Ferroptosis in Hepatocellular Carcinoma Based on Bioinformatics Methods" was retracted in 2023. Reasons: signs of a paper mill; suspected computer-generated content; unreliable results or conclusions; concerns about the data.

Prognostic model was widely utilized to evaluate the survivorship of patients suffering from cancer. In this project, HCC patients were allocated into FRL signature different risk subgroups according to the median risk score. The Kaplan-Meier analysis showed significantly shorter survival times in the high-risk group. The signature was well predicted via ROC curves and calibration plots. Furthermore, compared with the clinicopathological variables, this signature had a higher prediction accuracy of the prognosis.

The GSEA enrichment analysis revealed that the high-risk group was enriched primarily in glutathione metabolism, pathways in cancer, and other immune-related pathways. Depletion of glutathione (GSH) is a typical biochemical feature of ferroptosis [41]. Moreover, the enrichment of many immune-related biological pathways and functions further suggested that the tumor immunity had a close association with ferroptosis, or ferroptosis may affect the progress of HCC through immune mechanism. The subsequent ssGSEA results showed that the high-risk group had more aDCs (activated dendritic cells), macrophages, and regulatory T cells (Tregs). A recent study elucidated that activated dendritic cells are more abundant in patients with HCC, the mechanism may be that environmental semimature dendritic cells in HCC will activate Fc*γ*RIIlow/− B cells, thereby suppressing the function of cytotoxic T cells. At the same time, these semimature dendritic cells may also promote Tregs production and thus mediate immune tolerance [42]. Tumor-associated macrophages could produce cytokines and chemokines that inhibit antitumor immunity as well as propel cancer progression [43]. And the high infiltration of Tregs can also be used as an indicator of poor prognosis [44]. For B cells and mast cells, the proportion was smaller in high-risk group. Poor patient prognosis was found to be closely associated with a decline in tumor-infiltrating B cells [45]. The proportion of activated mast cells in tumors of HCC patients is much lower than in paraneoplastic tissues and even lower than in healthy people [46]. In addition, higher risk scores were linked to reduced antitumor immunity, such as an increase in MHC class I and a decrease in type II IFN response [47, 48]. Furthermore, the immune checkpoint scores were generally increased in the high-risk group, which could be related to the fact that liver cancer cells can utilize the activated immune checkpoint pathway to evade the recognition of the immune system, thus promoting the deterioration of tumors [49]. It can be inferred that the poor prognosis of high-risk HCC patients is related to elevated tumor immune escape. Meanwhile, drug sensitivity analysis suggested that chemotherapeutic drugs cisplatin, gemcitabine, imatinib, and paclitaxel were more sensitive in high-risk individuals. Therefore, ferroptosis-related lncRNAs can help patients choose more effective immunotherapy and chemotherapy and further provide a basis for personalized and accurate treatment of HCC patients.

The article "Prediction of Prognosis and Molecular Mechanism of Ferroptosis in Hepatocellular Carcinoma Based on Bioinformatics Methods" was retracted in 2023. Reasons: signs of a paper mill; suspected computer-generated content; unreliable results or conclusions; concerns about the data.

Undoubtedly, this study have some limitations. First of all, this is retrospective research using data from the TCGA database; thus, there may be some discrepancies. Secondly, the prognostic predictive signature must be confirmed by additional independent cohorts to demonstrate its stability. Finally, more experiments are required to discover the potential mechanisms of FRLs in HCC, which has not been confirmed by functional experiments to be related to HCC prognosis.

## 5. Conclusions

In summary, the establishment of five-FRL risk signature can be used as an independent predictor of prognosis in HCC patients. This lays the foundation for further investigation into the potential mechanism and clinical impact of FRLs in HCC.

## Figures and Tables

**Figure 1:** Flowchart of the study.

**Figure 2:** Identification of 84 DEFRGs in HCC tissues. (a) The volcano plots. (b) The heatmaps. (c) The boxplot. The red, black, and blue dots represent the upregulated genes, no difference, and downregulated genes, respectively; N: normal tissues; T: tumor tissues.

**Figure 3:** Construction of prognostic five-FRL signature. (a) Relative expression levels of five FRLs in HCC and normal tissues in TCGA. (b) The coexpression network of the five FRLs. (c) The Sankey diagram showed the connection degree between the five FRLs and FRGs. (d) The heatmaps of the five FRLs in different risk groups. (e) The Kaplan-Meier curves for the OS in different risk groups. (f and g) The number and survival status of patients in different risk groups. (h) ROC curves showed at the predictive efficiency of the risk signature for 1-, 3-, and 5-year survival.

The article "Prediction of Prognosis and Molecular Mechanism of Ferroptosis in Hepatocellular Carcinoma Based on Bioinformatics Methods" was retracted in 2023. Reasons: signs of a paper mill; suspected computer-generated content; unreliable results or conclusions; concerns about the data.

**Figure 4:** Relationship between variables in risk signature and clinical characteristics. (a and b) Relationship between risk score and survival outcome and tumor N stage. (c–f) Relationship between AC015908.3 and survival outcome, gender, tumor stage, and tumor T stage. (g and h) Relationship between LINC01138 and survival outcome and grade. (i–l) Relationship between LUCAT1 and survival outcome, gender, tumor M stage, and tumor N stage. (m and n) A forest plot of UniCox and multiCox analysis in the TCGA cohort. (o) ROC curves of the signature and clinicopathologic factors for OS.

**Figure 5:** Construction and verification of a nomogram. (a) Survival nomogram including clinicopathological factors and risk scores for 1-, 3-, and 5-year survival of HCC patients. (b–d) The calibration curve for predicting HCC patient survival at 1, 3, and 5 years in the TCGA cohort.

**Figure 6:** Internal verification of the five-FRL signature. (a and b) The Kaplan-Meier curves of the two cohorts. (c and d) ROC curves and AUCs at 1-, 3-, and 5-years survival of the two cohorts.

**Figure 7:** External verification of the five-FRL signature based on the GEO dataset. (a) The Kaplan-Meier curves of OS in different risk groups based on GSE76427. (b) ROC curves and AUCs at 1-, 3-, and 5-years survival based on GSE76427.

**Figure 8:** PCA maps based on different groupings of patients with high- and low-risk score. (a) Patient distribution based on whole genome. (b) Patient distribution based on FRG sets. (c) Patient distribution based on FRLs. (d) Patient distribution based on predictive signature. Patients in red are at high risk, while those in green are at low risk.

**Figure 9:** Results of enrichment analysis of GSEA.

**Figure 10:** Immune infiltration and immune checkpoints analysis in the low- and high-risk groups. (a and b) The boxplots of immune cell scores and immune function scores. (c) The expression of immune checkpoints among different risk groups. ns: not significant. ^∗^*P* < 0.05, ^∗∗^*P* < 0.01, and ^∗∗∗^*P* < 0.001.

**Figure 11:** Chemotherapy drug sensitivity analysis in the low- and high-risk groups. (a) Dasatinib. (b) Docetaxel. (c) Erlotinib. (d) Gefitinib. (e) Lapatinib. (f) Methotrexate. (g) Cisplatin. (h) Gemcitabine. (i) Imatinib. (j) Paclitaxel.

**Table 1:** Correlation between clinical variables and the five FRLs.

Id	AC015908.3	LINC01138	AC009283.1	Z83851.1	LUCAT1	Risk score
Fustat (vital status: alive = 0, dead = 1)	5.095 (1.133e-06)	-3.25 (0.002)	1.672 (0.097)	-1.556 (0.122)	-2.153 (0.034)	-3.16 (0.002)
Age (≤60 = 0, >60 = 1)	-0.299 (0.766)	0.726 (0.469)	1.416 (0.158)	0.063 (0.950)	-1.939 (0.054)	-0.566 (0.572)
Gender (female = 0, male = 1)	-2.376 (0.019)	0.393 (0.695)	-0.517 (0.606)	-1.49 (0.139)	-2.608 (0.010)	-1.672 (0.096)
Grade (grade 1 and 2 = 0, grades 3 and 4 = 1)	-0.123 (0.902)	-3.156 (0.002)	-1.287 (0.200)	-0.233 (0.816)	-1.802 (0.073)	-1.791 (0.076)
Stage (stages I and II = 0, stages III and IV = 1)	3.967 (1.222e-04)	-0.96 (0.339)	0.988 (0.325)	0.261 (0.794)	-0.037 (0.971)	-0.221 (0.825)
T (T1 and T2 = 0, T3 and T4 = 1)	3.597 (4.68e-04)	-0.934 (0.352)	1.042 (0.299)	0.491 (0.624)	-0.172 (0.864)	-0.277 (0.782)
M (M0 = 0, M1 = 1)	0.432 (0.707)	0.086 (0.939)	1.78 (0.213)	-0.766 (0.519)	5.005 (0.001)	0.106 (0.923)
N (N0 = 0, N1 = 1)	2.876 (0.097)	-1.136 (0.372)	-1.284 (0.325)	-1.033 (0.408)	5.363 (5.975e-04)	2.577 (0.017)

∗Assign categories to 0 and 1 for statistical analysis.

The article "Prediction of Prognosis and Molecular Mechanism of Ferroptosis in Hepatocellular Carcinoma Based on Bioinformatics Methods" was retracted in 2023. Reasons: signs of a paper mill; suspected computer-generated content; unreliable results or conclusions; concerns about the data.

**Table 2:** Patients' clinical characteristics in TCGA and GSE76427.

Variables	Training dataset	Validation cohort		
		Two random internal verification cohorts		GSE external verification cohort
	TCGA dataset (*n* = 343)	First cohort (*n*1 = 171)	Second cohort (*n*1 = 172)	GSE7642 dataset (*n* = 115)
Age				
≤60	165 (48.1%)	78 (45.6%)	87 (50.6%)	48 (41.7%)
>60	178 (51.9%)	93 (54.4%)	85 (49.4%)	67 (58.3%)
Gender				
Female	110 (32.1%)	49 (28.7%)	61 (35.5%)	22 (19.1%)
Male	233 (67.9%)	122 (71.3%)	111 (64.5%)	93 (80.9%)
Grade				
G1 + G2	214 (62.4%)	111 (64.9%)	103 (59.9%)	0 (0.0%)
G3 + G4	124 (36.2%)	59 (34.5%)	65 (37.8%)	0 (0.0%)
Unknown	5 (1.5%)	1 (0.6%)	4 (2.3%)	115 (100.0%)
Stage				
I + II	238 (69.4%)	117 (68.4%)	121 (70.3%)	90 (78.3%)
III + IV	83 (24.2%)	42 (24.6%)	41 (23.8%)	24 (20.9%)
Unknown	22 (6.4%)	12 (7.0%)	10 (5.8%)	1 (0.8%)
T				
T1 + T2	252 (73.5%)	126 (73.7%)	126 (73.3%)	0 (0.0%)
T3 + T4	88 (25.7%)	45 (26.3%)	43 (25.0%)	0 (0.0%)
Unknown	3 (0.9%)	0 (0.0%)	3 (1.7%)	115 (100.0%)
M				
M0	245 (71.4%)	126 (73.7%)	119 (69.2%)	0 (0.0%)
M1	3 (0.9%)	2 (1.2%)	1 (0.6%)	0 (0.0%)
Unknown	95 (27.7%)	43 (25.1%)	52 (30.2%)	115 (100.0%)
N				
N0	239 (69.7%)	120 (70.2%)	119 (69.2%)	0 (0.0%)
N1	3 (0.9%)	3 (1.8%)	0 (0.0%)	0 (0.0%)
Unknown	101 (29.5%)	48 (28.1%)	53 (30.8%)	115 (100.0%)

**Table 3:** Main characteristics of the previous related studies.

Authors	Year	Database	Sample size		FRL signature	AUC	
			Training cohort	Testing cohort		Training cohort	Testing cohort
Huang et al. [28]	22021	TCGA	218	145	AC009005.1, AC092119.2, AC099850.3, AL356234.2, GDNF-AS1, LINC01224, LUCAT1, and ZFPM2-AS1	0.719 (3 years)	0.745 (3 years)
Xu et al. [29]	2021	TCGA/GSE40144	255	59	CTD-2033A16.3, CTD-2116N20.1, CTD-2510F5.4, DDX11-AS1, LINC00942, LINC01224, LINC01231, LINC01508, and ZFPM2-AS1	0.812, 0.846, and 0.908 (3, 5, and 10 years)	0.635 (3 years)
Liang et al. [17]	2021	TCGA/GSE14520	374	488	RHPN1-AS1, MAPKAPK5-AS1, and PART1	0.711, 0.649, and 0.632 (1, 3, and 5 years)	0.711, 0.671, and 0.649 (1, 3, and 5 years)
Z. Zhang et al. [30]	2022	TCGA	206	136	PRRT3-AS1, LNCSRLR, MKLN1-AS, LINC01224, LINC01063, and POLH-AS1	0.812, 0.758, and 0.709 (1, 3, and 5 years)	0.845, 0.787, and 0.700 (1, 3, and 5 years)
Chen et al. [31]	2021	TCGA	174	174	AC245297.3, MYLK-AS1, NRAV, SREBF2-AS1, AL031985.3, ZFPM2-AS1, AC015908.3, and MSC-AS1	0.830 (1 years)	0.806 (1 years)
Wang et al. [32]	2021	TCGA/GSE76427	370	Not available	LUCAT1, AC099850.3, AL365203.2, AL031985.3, and AC009005.1	0.772, 0.707, and 0.666 (1, 3, and 5 years)	Not available

The article "Prediction of Prognosis and Molecular Mechanism of Ferroptosis in Hepatocellular Carcinoma Based on Bioinformatics Methods" was retracted in 2023. Reasons: signs of a paper mill; suspected computer-generated content; unreliable results or conclusions; concerns about the data.

## Data Availability

The data used to support the findings of this study are available from the corresponding author upon request.

## Supplementary Materials

Supplementary Materials Supplementary Table S1: 259 ferroptosis-related genes were downloaded from FerrDb database. Supplementary Table S2: 764 ferroptosis-related lncRNAs. Supplementary Table S3: 93 ferroptosis-related lncRNAs, which were substantially associated with the prognosis of HCC. Supplementary Table S4: results of sensitivity analysis of 138 chemotherapeutic drugs. Supplementary Figure 1: results of KEGG and GO analyses of 84 DEFRGs.
